This article has been retracted.

# Distribution and association between environmental and clinical isolates of *Cryptococcus neoformans* in Bogotá-Colombia, 2012-2015

**DOI:** 10.1590/0074-02760160201

**Published:** 2016-10-03

**Authors:** Norida Vélez, Patricia Escandón

**Affiliations:** Grupo de Microbiología, Instituto Nacional de Salud, Bogotá, Colombia

**Keywords:** Cryptococcus neoformans, cryptococcosis, environment, Colombia

## Abstract

The propagules of the fungal species *Cryptococcus neoformans* and *C. gattii*, whose varieties are distributed world wide, are the primary cause of cryptococcosis, a life threatening disease. The study of environmental and clinical isolates of *Cryptococcosis* is an important contribution to the epidemiology and ecology of the fungus. The aim of this work was to determine the presence of *C. neoformans* and *C. gattii* in the environment in Bogotá, Colombia’s capital city and to establish the relation between clinical and environmental isolates in the period 2012-2015. From a total of 4.116 environmental samples collected between October 2012 - March 2014, 35 were positive for *C. neoformans* var. *grubii*. From 55 cryptococcosis cases reported in Bogotá during 2012-2015, 49 isolates were recovered. From those, 94% were identified as *C. neoformans* var. *grubii* molecular type VNI; 4% as VNII and 1,2% as *C. neoformans* var *neoformans* VNIV. The 84 detected clinical and environmental isolates studied had a similarity between 49-100% according with molecular typing. The correlation between environmental and clinical samples confirms the hypothesis that patients acquire the disease from environmental exposure to the fungal propagules.

Cryptococcosis is an opportunistic mycoses of immunosuppressed and immunocompetent patients. Infection is acquired by inhalation of fungal propagules through environmental exposure. It is considered a potentially fatal infection of the lungs and the central nervous system (CNS). The etiological agents are *Cryptococcus neoformans* and *C. gattii*, whose varieties have a worldwide distribution. However, a recently proposed taxonomy for these species suggests there are seven species in the complex (Cabral 1999, Cogliati 2013, Hagen et al. 2015).

There are two varieties of *C. neoformans* mainly associated with HIV/AIDS patients, var. *grubii* (serotype A), distributed worldwide and var. *neoformans* (serotype D) that together with the hybrid AD, are concentrated in Europe (Viviani et al. 2006, Trilles et al. 2008, Heitman et al. 2011). These species have been isolated mostly from bird excreta, especially from pigeon, and decaying wood from different trees, except for the serotype D (Rosario et al. 2008, Trilles et al. 2008, Francis et al. 2013). Studies on the environmental distribution in different parts of the world have increased, such as in South Africa, Argentina, Brazil, India and Thailand (Ergin et al. 2004, Kuroki et al. 2004, Grover et al. 2007, Rosario et al. 2008, Trilles et al. 2008, Refojo et al. 2009). *C. gattii* is grouped into serotypes B and C, distributed in tropical, subtropical and template regions (Byrnes et al. 2009, Cogliati 2013), and affecting mostly immunocompetent persons. This species has been recovered from plant debris in trees like *Eucalyptus sp*, *Terminalia catappa*, *Corymbias*, among others. *C. gattii* has been reported in recent years in Australia, Italy, Spain, Netherlands, Japan, India, Colombia and South Korea (Granados & Castañeda 2006, Grover et al. 2007, Hagen & Boekhout 2010, Escandón et al. 2010, Colom et al. 2012, Hagen et al. 2012, Cogliati 2013).

In Colombia, environmental studies have reported isolates of *C. neoformans* var. *grubii* (serotype A) and *C. gattii* (serotype B and serotype C) from plant debris in trees like *Eucalyptus sp*, *T. catappa*, *Corymbias* and *Ficus*, and described that serotypes A and B were the most prevalent (Castañeda & Castañeda 2001, Granados & Castañeda 2005, Quintero et al. 2005, Escandón et al. 2010). In Bogotá, studies reported *C. neoformans* and *C. gattii* from 192 environmental and clinical samples, being serotype A the most prevalent, followed by serotype B and C (Ordoñez & Castañeda 1994).

In 2001, Castañeda and Castañeda (2001) described the association between *Cryptococcus* and *Eucalyptus* from a local park in Bogotá, with a positivity of 4% during a two-year sampling period. In 2005, Granados and Castañeda (2005) collected 480 environmental samples with a positivity of 7.9% for *C. neoformans* and, in 2010, Escandón et al. (2010) found a positivity of 11.7% for *C. gattii* isolated from *Corymbia ficifolia* in Bogotá.

A number of molecular typing techniques have been used to study the molecular epidemiology of *C. neoformans* and *C. gattii* (Meyer et al. 2003), providing more discriminatory power than conventional techniques (Perfect et al. 1993). Using polymerase chain reaction (PCR) fingerprinting, eight major molecular types have been established (Meyer et al. 2003). The major molecular types VNI and VNII correspond to *C. neoformans* var. *grubii*, being VNI the most prevalent in environmental and clinical isolates (Springer & Chaturvedi 2010, Cogliati 2013), VNIII corresponds to the AD hybrid and VNIV (Serotype D) corresponds to *C. neoformans* var. *neoformans*, found mainly in Europe (Viviani et al. 2006).

Molecular types VGI, VGII, VGIII and VGIV correspond to *C. gattii*, whose environmental and clinical distribution vary according to the region. It has been reported that molecular type VGI is the most frequent in Australia (Meyer et al. 2003); VGII in Canada, South America and Australia (Byrnes et al. 2009, Cogliati 2013), being the unique to report of an outbreak in Vancouver Island and in the North of USA (Byrnes et al. 2009); VGIII is most frequently recovered in South America (Meyer et al. 2003) and VGIV in South Africa and India (Springer & Chaturvedi 2010, Cogliati 2013).

In the last report of the Colombian Group for the Study of cryptococcosis, the annual incidence rate was 3.3x10^3^ cases in AIDS patients and in the general population 2.4x10^6^, between 2006-2010. This passive surveillance is important for the study of this opportunistic infection in AIDS patients, considered a sentinel marker for HIV infection (Escandón et al. 2012). The aim of this work was to determine the presence of *C. neoformans* and *C. gattii* in the environment in Bogotá and to establish the genetic relation of these isolates with those causing cases of cryptococcosis reported during the period 2012-2015.

## MATERIALS AND METHODS

*Study design* - Epidemiological and molecular study from environmental and clinical isolates in the capital city Bogotá - Colombia.

*Study area* - Bogotá is the capital of Colombia, located at 4º34 N latitude, 74º00 W longitude, and 2.630 meters above sea level, with an average temperature of 13.8ºC. A total of 15 areas were chosen and divided in six zones from north to south in Bogotá. Four areas previously determined to be positive (Granados & Castañeda 2005, Escandón et al. 2010) were included, and the others were chosen due to a high density of trees (Fig. 1).

**Fig. 1:** : description of the sampled areas for the recovery of *Cryptococcus neoformans*, recovered between October 2012 and March 2014 in the capital city of Colombia, Map of Bogotá with the six zones.

*Clinical isolates* - Information on cryptococcosis cases was gathered retrospectively from a passive surveillance during 2012-2015 from patients residing in Bogotá.

*Environmental sampling* - The methodology used for sampling was described by Escandón et al. (2010). Environmental samples from the hollows, leaves, bark, flowers, soil and fruits of two tree species, *Eucalyptus* sp. and *Corymbia* sp., were collected during every month between September 2012 and March 2014 (n = 19 months), in the selected areas previously described. A longitudinal sampling was carried out in those positive areas for a period of five months from October 2013 - March 2014.

*Environmental data* - Temperature, relative humidity, precipitation and sunshine in Bogotá during the study period were obtained from the Institute of Hydrology, Meteorology and Environmental Studies (http://www.ideam.gov.co.).

*Conventional techniques* - Environmental samples were identified by streaking onto Niger-seed agar as described by Granados and Escandón (Granados & Castañeda 2006, Escandón et al. 2010). Phenotypic tests were used for sample processing and confirmation of isolates as previously described (Kwon-Chung et al. 1982). DNA was extracted as reported by Escandón et al. (2006) and molecular type was determined by PCR fingerprinting with the unique primer (GTG)_5_ and restriction fragment length polymorphism (RFLP) of the *URA5* gene (Meyer et al. 2003, Escandón et al. 2010). PCR products were compared with reference strains reported and provided by Meyer et al. (2003).

The analysis of molecular types generated by PCR-(GTG)_5_ was performed using the Gel Compare 2® V.4.0 (Applied Maths, Sint-Martens Latem, Belgium) program. The Dice coefficient was used to compare the molecular types and establish genetic relationships between isolates. Clustering was based on the Unweighted Pair Group Method (UPGMA) algorithm with a tolerance 4.0% and optimisation of 1,5%.

## RESULTS

*Environmental samples* - Out of 4.116 environmental samples collected from *Corymbia sp* and *Eucalyptus sp* in Bogotá from six different zones (Fig. 1), 35 samples were positive for *C. neoformans* (0.9%). Of these positive samples, 20 (57.1%) were from bark, 13 (37.1%) from soil and two (5.8%) from fruit (Table I). From the positive samples, 110 colonies were recovered all belonging to *C. neoformans* var. *grubii*. *C. gattii* was not recovered.

**TABLE I:** Description of positive samples for *Cryptococcus neoformans* recovered between October 2012 and March 2014 in the capital city of Colombia, according to the type of tree and type of sample

			*Corymbia* sp	*Eucalyptus*			
				
Zones	Places	Total of samples	Bark	Bark	Fruit	Soil	Total
Zone 1	Av 19 - 105	4	0	0	0	0	0
	Parque 104 - Terpel	165	0	2	0	0	2
	Parque 106	10	0	0	0	0	0
Zone 2*	Bavaria	3	0	0	0	0	0
	Museo Chico	26	0	0	0	0	0
	Kra 7 entre 97 - 94	190	0	1	1	3	5
Zone 3*	Kra Once	707	1	0	0	0	1
	Cachivaches 85 - 105	21	0	0	0	0	0
	Virrey	26	0	0	0	0	0
Zone 4*	Gobernación	801	1	1	0	2	4
	Maloka	1027	0	14	0	7	21
Zone 5*	Parque de los Novios	184	0	0	1	1	2
	Universidad Nacional	922	0	0	0	0	0
Zone 6	Candelaria	26	0	0	0	0	0
	Plaza de Bolívar	4	0	0	0	0	0
Total		4116	2	18	2	13	35

*: places which had been positive in previous studies.

Most of the positive samples (n = 27) were obtained in July and November 2013, coinciding with previous periods of high precipitation. Only few samples (n = 8) were recovered during the dry season temperature and relative humidity was relatively constant throughout the study period with no other obvious associations (Fig. 2).

**Fig. 2:** : positive isolates of *Cryptococcus neoformans* and climatic parameters: precipitation (mms) and sunshine (h).

*Description of clinical cases of cryptococcosis* - A total of 55 surveys were received during the study period, corresponding to new cases of cryptococcosis, reported mainly in men (43 cases, 78.2%). Patients aged 16-79 years old were the most affected (59.3% of the cases with a median of 43 years). The main risk factor was HIV infection in 36 (65.5%) cases, other risk factors were diabetes and leukemia and chronic renal failure. One patient presented with autoimmune disease (lymphoma) (Table II).

**TABLE II:** Clinical manifestations, pharmacological treatment and diagnosis of Cryptococcosis cases in Bogotá, Colombia (2012-2015)

Characteristics	(n)	(%)
Sex		
Male	43	78.2
Female	12	21.8
Clinical features		
Headache	45	81.8
Fever	28	50.9
Nausea and vomiting	21	38.2
Confusion	18	32.7
Loss weight	17	30.9
Seizures	13	23.6
Meningeal signs	7	12.7
Cough	13	23.6
Visual alterations	8	14.5
Risk factors		
HIV infection	36	65.5
Corticosteroids	4	9.1
Autoimmune disease	1	
Diabetes	1	5.4
Others (leukemia, CT)	2	
No risk factor	11	20
Type of diagnosis		
Positive Culture(one strain was not viable)*	27	49.1
Positive Culture and Antigen	2	3.6
Positive Culture and direct examination	17	31.0
Positive Culture, direct examination and Antigen	4	7.3
Direct examination	2	3.6
Direct examination and antigen	3	5.4
Total	55	100
Type of antifungal used		
Amphotericin B	26	47.3
Fluconazole	3	5.5
Combined	0	0
No theraphy	26	47.3

*: it was not possible to recover the strain.

The most common clinical manifestations are described in Table II, consisting mostly of headache and fever.

From the patients, 47.2% were treated with antifungal agents, with amphotericin B being the most common antifungal used (47.3%), followed by fluconazole (5.5%). Neurocryptococosis was the most common clinical form of the disease. Laboratory diagnosis was performed using the conventional methods of direct examination, antigenemia and culture. In 49/55 cases, the isolate was recovered; in six cases it was not possible to recover the strain and only medical history is described (Table II).

*Molecular characterisation* - Molecular type determination revealed that from the 84 isolates characterised (n = 49 clinical and n = 35 environmental), 79 isolates (94%) were *C. neoformans* var. *grubii* molecular type VNI, 4 (4.8%) isolates VNII and 1 (1.2%) VNIV (Fig. 3).

**Fig. 3:** : characterisation of clinical and environmental isolates of *Cryptococcus neoformans* typed by GTG5-PCR fingerprinting (A) and RFLP-URA5 (B).

Of the two main groups identified, group I had a similarity of 48%, including isolates of *C. neoformans* var. *grubii* molecular type VNI and VNII. A subgroup of group 1 was identified, with an index of similarity between 50-100%, containing all isolates belonging to the molecular type VNI. In subgroup A, 10 genetically indistinguishable clusters were identified (with 100% similarity), containing five clusters of clinical and environmental isolates. Group II contained the only VNIV clinical isolate recovered and the control strain with a 100% similarity. Four clinical and one environmental isolates did not group with any of the other isolates (Fig. 4).

**Fig. 4:** : GTG5-PCR fingerprinting dendrogram of the *Cryptococcus neoformans* clinical and environmental isolates from Bogotá. Dendrogram of the PCR-fingerprint from clinical (♥)and environmental isolates (♦), Group (A), clinical and environmental isolations grouped with 100% similarity index. Software GelCompar II version 4.0, tolerance % and optimisation 1.5.

## DISCUSSION

In Colombia, several studies have been performed to describe the environmental importance of *Cryptococcus*, and the potential relation of environmental and clinical isolates. In some of these studies, isolates of serotypes A, B and C have been recovered, from different species of trees including *Eucalyptus* sp, *Ficus sp*, *C. ficifolia*, *T. catappa*, among others, similarly to the reports of other groups in countries like Brazil and India (Randhawa et al. 2001, Trilles et al. 2008).

*C. neoformans* var. *grubii* serotype A was the only species recovered in the environmental samples collected in this study, with a frequency of 0.7 %. This positivity falls within that of the literature, where a frequency between 0.1-69% has been reported, confirming the same results obtained in other environmental studies, and reinforcing the predominance of this species in the environment around the world (Perfect et al. 1993, Randhawa et al. 2001, Escandón et al. 2006, Trilles et al. 2008).

In this study we found *C. neoformans* in places with high density of trees, people and pigeons, distributed in the center and north-west of the city. In other studies of Bogotá, authors reported a positivity from the environment of 7.9% for *C. neoformans* (Granados & Castañeda 2005). The yeast was recovered in five out of the six studied areas, and from those, four were previously reported as positive in other studies (Escandón et al. 2006, Granados & Castañeda 2006), suggesting permanence and colonisation of the fungus over time. Additionally, a new area was identified as positive for *C. neoformans*.

In this study *C. gattii* was not recovered, from clinical nor environmental samples, which is in contrast to other studies reported in Bogotá were *C. gattii* was isolated in 11.72% from *C. ficifolia* samples (Escandón et al. 2010).

This study reinforces the predominance of *C. neoformans* in *Eucalyptus* tree species; as has been found in studies in Egypt (Cogliati 2013), Brazil (Trilles et al. 2008) and Australia (Ellis & Pfeiffer 1990). The preference of *C. neoformans* for this type of tree may be due to the specific characteristics of the wood, for example due to the hollows, as suggested by Ellis and Pfeiffer (1992).

The months when the fungus was recovered coincide with previous periods of high precipitation, confirming the findings reported by Granados and Castañeda (2005, 2006), who analysed the presence of *C. neoformans* in environmental samples and concluded that the fungus was most frequently recovered in the rainy season.

In Colombia, cryptococcosis by *C. neoformans* var. *grubii* has high morbidity and mortality, especially in HIV-positive patients in (Escandón et al. 2010, Lizarazo et al. 2014). Chronic lung disease, cancer and immune disorders such as neoplasia, HIV/AIDS, predispose patients to infection by *Cryptococcus* (Hull & Heitman 2002). The latter is apparent in Colombian patients, in which risk factors such as HIV infection, leukemia, diabetes and renal failure were presented (Escandón et al. 2010), as well as the predominance of *C. neoformans* var. *grubii* (serotype A) (98.1%). The finding in Colombia that var. *grubii* is the most common clinical isolate correlates with the reports from around the world, as well as the association of molecular type VNI with AIDS patients (Escandón et al. 2006).

Genotype VNI was identified in 94% of the environmental and clinical isolates, in agreement with the distribution reported in South America (Meyer et al. 2003), Vietnam (Chau et al. 2010), India (Jain et al. 2005), Malaysia (Tay et al. 2010), China (Feng et al. 2008), Korea (Choi et al. 2010) and frequently recovered in the environment (Jain et al. 2005, Cogliati 2013). Molecular studies found a relation between clinical and environmental isolates, reinforcing the hypothesis that infection is acquired by the inhalation of infectious propagules present in the environment (Meyer et al. 2003, Trilles et al. 2008, Byrnes et al. 2009, Velagapudi et al. 2009). In this study, clinical and environmental isolates were found to be between 48-100% similar. This is congruent with other studies around the world, such as the reported in 2008 by Trilles et al. (2008), who found a similarity index of 50% in VNI, being the most prevalent in 443 environmental and clinical isolates from Brazil. In the same year Meyer reported a similarity index of 50.4% between clinical and environmental isolates of *C. neoformans* var. *grubii* (Meyer et al. 2003).

The search of *C. neoformans* and *C. gattii* in the environment needs to be included as a routine practice, in those areas were cryptococcosis cases are prevalent, as a tool that will help us identify colonised areas which may represent increased exposure risks to the patients. The continuous finding of the fungus both in the environment and in the patients of the capital city of Colombia reinforces the need to direct our efforts into more active surveillance of the disease.

Ecological studies are relevant in the epidemiological study of this pathogen; therefore the continuity of clinical research is important for ecological studies, the results of which may allow us to determinate areas where the fungus can find favorable conditions to develop in Colombia.
